# MiR-144 Inhibits Uveal Melanoma Cell Proliferation and Invasion by Regulating c-Met Expression

**DOI:** 10.1371/journal.pone.0124428

**Published:** 2015-05-11

**Authors:** Lei Sun, Guangqing Bian, ZhaoJun Meng, Guangfu Dang, DeJing Shi, Shuyong Mi

**Affiliations:** 1 Department of Ophthalmology, The Fourth Hospital of Harbin Medical University, Harbin, 150001, Heilongjiang, China; 2 Department of Ophthalmology, Shandong Provincial Qianfoshan Hospital, Jinan 250000, Shandong, China; Peking Union Medical College Hospital, CHINA

## Abstract

MicroRNAs (miRNAs) are a group endogenous small non-coding RNAs that inhibit protein translation through binding to specific target mRNAs. Recent studies have demonstrated that miRNAs are implicated in the development of cancer. However, the role of miR-144 in uveal melanoma metastasis remains largely unknown. MiR-144 was downregulated in both uveal melanoma cells and tissues. Transfection of miR-144 mimic into uveal melanoma cells led to a decrease in cell growth and invasion. After identification of two putative miR-144 binding sites within the 3' UTR of the human c-Met mRNA, miR-144 was proved to inhibit the luciferase activity inMUM-2B cells with a luciferase reporter construct containing the binding sites. In addition, the expression of c-Met protein was inhibited by miR-144. Furthermore, c-Met-mediated cell proliferation and invasion were inhibited by restoration of miR-144 in uveal melanoma cells. In conclusion, miR-144 acts as a tumor suppressor in uveal melanoma, through inhibiting cell proliferation and migration. miR-144 might serve as a potential therapeutic target in uveal melanoma patients.

## Introduction

Uveal melanoma, including choroidal and iris melanomas, is one of the most common types of primary intraocular malignancy, with an estimated annual incidence of ~5.1 cases per million[1, 2]. Uveal melanoma has a high rate of metastasis, mainly spreading hematogenously to liver[3, 4]. Early metastasis contributes to the high mortality rate of uvealmelanoma[5, 6]. Although major advances have been made in the diagnosis and therapy of uveal melanoma, the 5-year relative survival rate has not improved from 1973 to 2008, especially in patients with metastatic disease[7]. Since the molecular mechanisms of its aggressiveness remain not elucidated, no therapy is effective for metastatic uveal melanoma patients[8, 9]. Therefore, understanding the crucial signals that contribute to the invasive and metastatic potential of uveal melanoma might help to identify novel therapies for uveal melanoma patients.

MicroRNAs (miRNAs) are small (19–24nt), single stranded, noncoding RNAs, which can regulate gene expression posttranscriptionally[10–13]. Through binding to specific target mRNA, mature miRNAs can trigger mRNA degradation, stability or inhibition of translation[14–17]. Increasing evidences have shown that miRNAs play crucial roles in many biological processes, such as cell proliferation and apoptosis, glucose and lipids metabolism, signal transduction and responses[18–23]. In addition, miRNAs participate in human tumor genesis, which could add new insights into understanding the mechanisms of human malignancies[24, 25]. Aberrant miRNA expression is proved to associate with various human cancers, functioning as oncogenes or tumor suppressors [26–30].

In our study, miR-144 was down-regulated in uveal melanoma cells and tissues. Ectopic expression of miR-144 could inhibit uveal melanoma cell proliferation and invasion in vitro. Moreover, c-Met was identified as the potential targets of miR-144, and miR-144 might suppress tumor growth and invasion by repressing the expression of c-Met. Our findings suggest that miR-144 may function as a novel tumor suppressor gene in uveal melanoma and can be a potential therapy target for uveal melanoma.

## Materials and Methods

### Ethics statement

All patients were written informed consent in our study. Our study was approved by the Medical Ethics Committee of The Fourth Hospital of Harbin Medical University.

### Samples collection and cell culture

Five tumor samples were collected from primary uveal melanomas patients and immediately frozen in liquid nitrogen. Tumor samples were stored at liquid nitrogen. Normal uveal samples were obtained from the Beijing Tongren Eye Bank (Beijing, China). The uveal melanoma cell lines (MUM-2B, C918, MUM-2C and OCM-1A) and the human melanocyte cell line (D78) were obtained from the Cell Bank of the Chinese Academy of Sciences (Beijing, People’s Republic of China). The OCM-1A and MUM-2C cells were cultured in Dulbecco’s modified Eagle’s medium (DMEM), which were supplemented with 10% fetal bovine serum (FBS) and MUM-2B, C918 in RPMI 1640 supplemented with 10% FBS.

### qRT-PCR

Total RNA was isolated from frozen specimens (or the cells) using Trizol (Invitrogen). To measure the expression of miR-144, RNA (2μg) was used by quantitative RT-PCR (qRT-PCR) with the TaqMan microRNA assays reverse transcription kit according to manufacturer’s instructions (Applied Biosystems, Foster City, CA). U6 was used as internal control. Real-time PCR was performed with of cDNA (1mL) on Real-Time PCR System (Applied Biosystems, Foster City, CA) in duplicates. −ΔCT ^CT^ represents the difference of CT values between internal control and miR-144. ΔΔCT was used to present the difference of ΔCT values between paired specimens. 2^ΔΔCT^ means the exponential value of ΔCT, representing fold change in expression (S1 Table).

### Cell proliferation

Cell proliferation was examined by the Cell Counting Kit-8 (CCK-8; Dojindo, Kumamoto, Japan) assay, in accordance to manufacturer’s instructions. Absorbance was detected at 450 nm and measured by Quant Universal Microplate Spectrophotometer (BioTek Instruments, Inc.).

### Oligonucleotide transfection

The miR-144 inhibitors, mimics and their controls were synthesised from GenePharma (Shanghai, China). Cells were transfected with them to a final oligonucleotide concentration at20 nmol/L. Cell transfection processes were done by Lipofectamine 2000 (Invitrogen) following to the instructions.

### Cell invasion assays

The transwell chambers were incubated to solidify with Matrigel (BD Biosciences, San Jose, CA, USA) at 37°C for 6 h. 4×10^5^ cells were suspended in serum-free DMEM which added into the upper chamber after 24 h, and medium containing 10% FBS was put to the lower chamber. After 24 h, invasive cells on the lower chamber were stained and counted.

### Western blot

Total protein was isolated from frozen tissues (or the cells) using Protein Extraction Kit (KeyGen, Nanjing, China). Proteins were separated using 10% SDS-PAGE and then transferred to PVDF membrane, which was incubated with the antibody for c-Met (Sigma, St. Louis, MO) or GAPDH (Cell Signaling Technology, Beverly, MA, USA). The membrane was washed and incubated with HRP-conjugated secondary antibody. Intensity of the bands was measured using the enhanced chemiluminescence (ECL, Amersham Pharmacia Biotech) system and subsequently exposed.

### Luciferase assay

MUM-2B cells were seeded in 24-well plates (1×10^5^ cells/well) for 24 hours. For the reporter gene assay, cells were cotransfected with pGL3-c-Met-3’UTR (0.5μg) or pGL3-c-Met-3’UTR mut plasmid, the phRL-SV40 control vector (0.05 ng, Promega, USA), and miR-144 mimic or scramble by Lipofectamine 2000 (Invitrogen, USA). The firefly and renilla luciferase activities were measured using the dual luciferase assay (Promega, USA) 24 hours after transfection.

### Statistical analysis

Data was presented as mean ±SD. The differences between two groups were used Student’s t-test and the differences in more than two groups were used A one-way analysis of variance (ANOVA). All statistical analyses were performed using SPSS 16.0 (SPSS Inc., USA). P<0.05 was considered as statistically significant.

## Result

### MiR-144 was decreased in uveal melanoma cells and tissues

qRT–PCR analysis showed that the expression of miR-144 was decreased in uveal melanoma cell lines (MUM-2B, C918, MUM-2C and OCM-1A) compared with D78, human melanocyte cell line(Fig 1A). In addition, miR-144 was also decreased in human uveal melanoma tissues compared with normal uvea tissues (Fig 1B).

**Fig 1:** The expression ofmiR-144 was downregulated in uveal melanoma cells and tissues (A) qRT–PCR analysis of miR-144expression in uveal melanoma cell lines (MUM-2B, C918, MUM-2C and OCM-1A) and one human melanocyte cell line (D78). The level of miR-144 expression was normalized to U6. (B) qRT–PCR analysis of miR-144expression in 5human uveal melanoma tissues and 5 normal uvea tissues. The level of miR-144 expression was normalized to U6.***p<0.001.

### Overexpression of miR-144inhibited proliferation and invasion of uveal melanoma cells

The expression of miR-144 was increased in MUM-2B cells transfected with miR-144 mimics, and decreased in cells transfected with miR-144 inhibitor (Fig 2A). The growth rate was reduced in MUM-2B cells transfected with miR-144 mimics compared with cells transfected with scramble mimics (Fig 2B). Meanwhile, miR-144 inhibitor promoted the MUM-2B cells proliferation (Fig 2B). The invasiveness of cells was decreased in cells transfected with miR-144 mimics compared with the scramble group and control group cells and increased in cells transfected with miR-144 inhibitor compared with the scramble group and control group (Fig 2C).

**Fig 2:** Overexpression of miR-144inhibited proliferation and invasion of uveal melanoma cells (A) qRT–PCR analysis of miR-144 expression in MUM-2B cells which was transfected miR-144 mimics, inhibitors, scramble or control. (B) The CCK-8 proliferation assay showed that miR-144 mimics can inhibit the proliferation of the MUM-2B cells. Meanwhile, miR-144 inhibitor increased the proliferation of the MUM-2B cells. (C) Invasion analysis of MUM-2B cells after treatment withmiR-144 mimics, inhibitors or scramble or control; the relative ratio of invasive cells per field is shown below, *p<0.05, ** p<0.01, and ***p<0.001.

### c-Met is a critical downstream target of miR-144

Analysis using available algorithms suggested that c-Met was a potential target gene of miR-144 (Fig 3A). Luciferase reporter gene assays demonstrated that miR-144 reduced luciferase activity of the c-Met wild-type reporter gene but not the mutant type, suggesting that miR-144 directly targeted the c-Met3’UTR (Fig 3B). The mRNA level of c-Met was decreased after transfection miR-144 mimics and increased after transfection miR-144 inhibitor (Fig 3C). The ability of miR-144 to regulate the expression of the c-Met was also verified by western blotting (Fig 3D).

**Fig 3:** c-Met is a critical downstream target of miR-144 (A) Targetscan analysis using available algorithms indicated that c-Met is a theoretical target gene of miR-144. (B) Luciferase reporter gene assays showed that ectopic of miR-144 remarkably reduced luciferase activity in the c-Met wild-type reporter gene but not the mutant c-Met 3’UTR.(C) qRT-PCR analysis of c-Met expression in the MUM-2B cells which was transected miR-144 mimics, inhibitors, scramble or control. GAPDH was used as internal control. (D) Western blot analysis has shown that miR-144 mimic inhibited the protein expression of c-Met in MUM-2B cells. GAPDH was also detected as a loading control. ***p<0.001.

### Downregulation of c-Met inhibits uveal melanoma cell proliferation and invasion

Western blotting analysis showed that siRNA-c-Met inhibited the expression of c-Met (Fig 4A). Downregulationof c-Met decreased proliferation and invasion of uveal melanoma cell. When miR-144 inhibitor and si-c-Met were cotransfected into MUM-2B cells, miR-144 inhibitor enhanced the si-c-Met-induced inhibition of proliferation and invasion in uveal melanoma cells (Fig 4B and 4C).

**Fig 4:** Inhibition of c-Met inhibits uveal melanoma cell proliferation and invasion (A) Western blotting analysis was performed to examine the effects of siRNA-c-Met on the expression of c-Met. GAPDH was also detected as a loading control. (B) The cell growth in MUM-2B cells co-transfected with either siRNA-c-Met, siRNA-c-Met and miR-144 inhibitor or control using CCK-8 proliferation assay. (C) The cell invasive in MUM-2B cells co-transfected with either siRNA-c-Met, siRNA-c-Met and miR-144 inhibitor or control using invasion assay. *p<0.05, ** p<0.01, and ***p<0.001.

### Restoration of miR-144 inhibits c-Met-mediated uveal melanoma cell proliferation and invasion

Western blotting analysis demonstrated that pCDNA-c-Met enhanced the expression of c-Met (Fig 5A). Overexpression of c-Met promoted cell proliferation and invasion in uveal melanoma. In addition, when miR-144 mimic and pCDNA-c-Met was cotransfected into MUM-2B cells, miR-144 mimic repressed the pCDNA-c-Met-induced proliferation and invasion in uveal melanoma cells (Fig 5B and 5C).

**Fig 5:** Restoration of miR-144 inhibits c-Met-mediated uveal melanoma cell proliferation and invasion (A) The protein expression of c-Met was detected using western blotting analysis. (B) The cell growth in MUM-2Bco-transfected with either miR-144 mimic and 2.0 μgpCDNA-c-Met or pCDNA empty vector using CCK-8 proliferation assay. (C) The cell invasive in MUM-2B cells co-transfected with either miR-144 mimic and 2.0 μgpCDNA-c-Met or pCDNA empty vector using invasion assay. *p<0.05, ** p<0.01, and ***p<0.001.

## Discussion

Emerging evidences have indicated that miRNAs have a crucial role in the pathogenesis of cancer through regulating genes involved in cell proliferation, migration, and invasion[15, 31–33]. Deregulation of miRNAs is common in cancers, where miRNAs might act as oncogene or putative tumor suppressor genes [34–36]. In the present study, miR-144 was downregulated in human uveal melanoma cells and tissues. Specifically, miR-144 inhibited cell proliferation and invasion. Target prediction and in vitro functional studies showed that c-Met was a direct target of miR-144. Importantly, miR-144 mimic rescued the c-Met-induced cell invasion and proliferation. These findings suggest that miR-144 has an important role in inhibiting the development and progression of uveal melanoma.

There is increasing reports on the role of miR-144 in carcinogenesis[37]. MiR-144 was originally identified as an erythroid-specific miRNA, which was required for subsequent urvival and maturation of the erythroid lineage[38]. Downregulation of miR-144 was found in various cancers, such as hepatocellular carcinoma, lung cancer, and osteosarcoma[39–41]. Akiyoshi et al. proved that miR-144 expression was inversely correlated with gastric cancer [42]. Sureban et al. also showed that knockdown of doublecort in and CaM kinase-like-1 (DCAMKL-1) increased miR-144 expression, which in turn inhibited epithelial-mesenchymal transition (EMT) of pancreatic cancer[43]. However, there are also contradictive reports. Zhang et al. showed that miR-144 promoted proliferation, migration, and invasion of nasopharyngeal carcinoma through repressing phosphatase and tensin homolog (PTEN)[44]. Thus the function of miR-144 in carcinogenesis seems to be complicated and highly tissue-specific. However, the role of miR-144 in uveal melanoma remains unclear. In our study, the expression of miR-144 was downregulated in human uveal melanoma cells and tissues. Moreover, introduction of miR-144 can reduceduveal melanoma cell proliferation and invasion. These results suggest that miR-144 might act as a tumor suppressor gene whose down-regulation contributes to the progression and metastasis of uveal melanoma.

MiRNAs control cellular functions by inhibiting the expression of genes; therefore, elucidation of their target gene is crucial. In the present study, for the first time, miR-144 was demonstrated to inhibit the proliferation and invasion of uveal melanoma cells by regulating the expression of c-Met. Activated MET oncoprotein, also known as c-MET, contribute to the tumorigenesis of a wide variety of cancers[45]. c-Met has a major influence on biological processes including cellular proliferation, migration and invasion[46]. Alterations of c-Met may play a role in tumorigenesis of many cancers such as gastric cancer, bladder cancer, and colorectal cancer[47–49]. Overexpression of c-Met is considered as a novel potential or even an independent predictor of poor prognosis for clinical patients[50]. Moreover, c-Met is overexpressed in 60% to 86% of solid tumors, and associated with tumor aggressiveness in uvealmelanoma[51, 52]. Previous study showed that c-Met played a crucial role in the spreading of uveal melanoma in a murine model of selective liver metastasis[53]. C-Met activation was observed in uveal melanoma through indirect gene activation[54]. In our study, c-Met enhanced uveal melanoma cell proliferation and invasion; inhibition of c-Met reduced the uveal melanoma cell proliferation and invasion. Restoration of miR-144 inhibited c-Met-mediated uveal melanoma cell proliferation and invasion. These results demonstrate that miR-144 may act as a tumor suppressor in uveal melanoma by targeting c-Met.

In conclusion, the present study demonstrated that miR-144 was downregulated in uveal melanoma tissues and cell lines. Ectopic expression of miR-144 inhibited uveal melanoma cell proliferation and invasion. Further investigation revealed that c-Met was a potential target of miR-144. Therefore, miR-144 may serve as a potential therapeutic target in uveal melanoma patients.

## Supporting Information

S1 Table Primer sequence. (DOCX)
